This article has been retracted.

# Design optimization of office building envelope by developed farmland fertility algorithm for energy saving

**DOI:** 10.1016/j.heliyon.2023.e23387

**Published:** 2023-12-07

**Authors:** Chunyuan Yang, Siyao Yu, Yi Cao, Sama Abdolhosseinzadeh

**Affiliations:** a College of Culture and Tourism, Qujing Normal University, Qujing 655011, Yunnan, China; b College of Design and Engineering, National University of Singapore, 21 Lower Kent Ridge Road, Singapore 119077, Singapore; c Anhui University of Finance and Economics, Anqing 246000, Anhui, China; d University of Mohaghegh Ardabili, Ardabil, Iran; e College of Technical Engineering, The Islamic University, Najaf, Iraq

**Keywords:** Developed farmland fertility algorithm, Energy saving, Building envelope, Construction expense, Meta-heuristic

## Abstract

This study focuses on designing sustainable buildings with a specific emphasis on reducing energy consumption and optimizing costs. To address the time-consuming nature of simulation software like TRNSYS and Energy Plus, a novel meta-heuristic optimization algorithm called the Developed Optimization Algorithm of Farmland Fertility (DFFA) is provided. The DFFA algorithm is utilized to optimize parameters related to the building envelope, encompassing walls, windows, and glass curtain walls, aiming to minimize energy demand and construction expenses. Comparative analysis with other approaches such as EPO, LOA, MVO, and FFA demonstrates significant reductions in energy consumption and building design costs achieved by employing the proposed algorithm. Furthermore, the DFFA algorithm yields the desired results within fewer iterations. By increasing the surface area of the glass curtain wall and total window space, improvements in natural ventilation and interior lighting are observed. Despite similar window opening measurements across the compared methods, the suggested algorithm surpasses others when it comes to overall cost and energy efficiency. The total cost reduction compared to the initial design amounts to 39 %. Thus, the DFFA algorithm proves to be more effective in conserving energy in buildings compared to other analyzed procedures. This research serves as a case study and presents a promising method applicable to designing various building types under different weather conditions in future projects.

## 1 Introduction

The limitations of energy resources and the increasing consumption, coupled with the excessive energy usage by different societies, along with environmental pollution and the wastage of national funds, have put the future of human life at risk [1]. Structures constitute a substantial portion of the total global consumption of energy. Therefore, a thorough analysis of buildings' energy performance is crucial [2]. To construct a building that places emphasis on energy efficiency, the first step involves understanding the appropriate methodology for designing it [3]. Furthermore, the most essential factors in minimizing heat gain in buildings are the building form, appropriate orientation on the site, building envelope systems, and building materials [4]. Buildings hold considerable untapped energy-saving potential.

Due to the increasingly critical conditions of global warming, green buildings and topics related to energy consumption reduction have garnered more attention worldwide [5]. It is essential to maximize energy efficiency and minimize costs in office buildings, considering the substantial amount of energy they consume [6]. The aim of constructing green buildings is to enhance the indoor environment, mitigate energy wastage from cooling and heating, and mitigate the adverse environmental impacts of construction [7]. The energy usage of green buildings can be significantly diminished by optimizing the structural shell [8]. The fundamental objective of a building envelope is to provide a physical barrier between the inside and outside surroundings, capable of withstanding water, light, air, and heat [9]. It can be stated that excellence within the building environment and energy effectiveness are significantly impacted by the building envelope [10]. The energy effectiveness of building envelopes is affected by various parameters, including weather conditions, window and glass area, orientation, window shading, wall, and ceiling insulation [11]. Therefore, the design of green buildings involves evaluating numerous combinations of these parameters [12].

### 1.1 Related works

Many works have been done in the field of building design optimization [13], and we will present some of them. Ugur Acar et al. [14] focused on raising the energy and financial efficiency of residential structures during the preliminary design stage by emphasizing the multi-purpose enhancement of building envelope variables in Turkey. In their study, the goals were defined as reducing the primary capital expense of the structure envelope and minimizing the overall thermal energy requirement. They implemented the developed code of the NSGA-II genetic algorithm in the MATLAB environment to present the solutions of the Pareto set for the two provinces under consideration. Finally, they compared the life cycle costs (LCC) of the solutions from the Pareto set after applying the envelope optimization approach. The conclusion illustrated that the suitable assortment of structural envelope parameters in the initial design phase greatly decreases the LCC.

Fabrizio Ascione et al. [15] presented a multi-criteria optimization method to lessen energy usage, thermal discomfort, and overall cost. They utilized a genetic algorithm by coupling Energy Plus with MATLAB®. The design variables included the radiative properties of plaster, set point temperature, thermophysical properties of envelope details, building orientation, and window types. After conducting a Pareto optimization, the genetic algorithm generated two optimal solutions: one that optimizes primary energy consumption (PEC) and another that minimizes the global cost associated with energy (GC). The presented approach was related to an apartment building in Italy. The conclusions presented provided valuable methods for the renovation of Italian residential buildings in terms of cost optimization and energy efficiency. The ideal outcomes yielded minimal amounts of PEC, ranging from 62.0 to 91.9 $kWhp/m^{2}a$, and GC, ranging from 456 to 665 $€/m^{2}$, depending on the location.

Mohammad Najjar et al. [16] developed an integrated optimization approach that combines building data design and life cycle assessment to create energy-efficient structures. They examined a mathematical optimization model that integrates BIM-LCA, and this integrated optimization process resulted in sustainable decisions for residential construction. The study showed that the annual energy consumption intensity and environmental impacts can be reduced by 45 % and 30 %, respectively.

Aiman Albatayneh [17] presented the optimization of building envelope parameters for a household dwelling located in the warm and semi-dry Mediterranean weather region of Amman. The objective was to decrease the heating and cooling burdens while ensuring thermal satisfaction through the application of mechanical heating and cooling systems [18]. The optimization process began with a simulation employing DesignBuilder software, subsequent to a sensitivity examination of twelve design parameters to assess their impact on heating and cooling demands. Finally, the optimization was carried out using a genetic algorithm. The ultimate findings demonstrated that the overall energy usage could be decreased to 293.74 kWh/year, in contrast to 5225.97 kWh/year for the standard unit.

Yuxing Wang and Chunyu Wei [19] introduced a superior design approach for the “office building facade using a quantum genetic algorithm. By optimizing the building's facade structure, including walls, windows, window quantity, glass curtain walls, etc., they aimed to reduce construction expenses while fulfilling the required energy standards. In their study, compared to traditional genetic algorithms, optimizing the layout of the office building's facade structure at the desired ENVLOAD value resulted in a 13.8 % rise in the total area of windows, a 14 % boost in the glass curtain wall ratio, and a 7 % decrease in costs. Furthermore, when compared to the initial design, the overall cost was decreased by 35.3 %.

Yukai Ke et al. [20] employed the Enhanced Crow Search Algorithm in tandem with the EnergyPlus simulation application to effectively fine-tune the energy consumption of an office place situated in four 4 distinct urban centers within Australia. The findings of the study indicate that the implementation of energy-saving measures resulted in a reduction in energy usage exceeding 11.8 %. Their proposed method demonstrated “exceptional performance compared to benchmark algorithms in relation to solution quality and computational economy.

### 1.2 Research gap

The incorporation of simulation technologies in evaluating energy consumption and financial implications related to building envelopes is crucial for precise analysis. However, current methodologies often require precise construction specifications, resulting in time-consuming computations. Additionally, these methodologies frequently overlook the vital interconnections between optimizing energy systems design and the building envelope's characteristics. Neglecting these interdependencies can lead to suboptimal designs and missed opportunities for energy efficiency and cost reductions. Therefore, the main goal of this study is to address these existing research gaps by introducing an innovative meta-heuristic optimization algorithm called the Developed Optimization Algorithm of Farmland Fertility (DFFA). Also, in this research, the main algorithm for Farmland Fertility Optimization has been developed through two new strategies, which improve the results compared to the use of the main algorithm.

### 1.3 Novelty

The main contribution and novelty of this study lie in two key aspects. Firstly, we propose the Developed Optimization Algorithm of Farmland Fertility (DFFA), a novel meta-heuristic optimization algorithm specifically designed for sustainable building design. This addresses a critical research gap by providing an efficient and effective solution for optimizing building envelope parameters. The DFFA algorithm aims to achieve significant reductions in energy consumption and building design costs by optimizing interdependent relationships between elements like walls, windows, and glass curtain walls. This specialized algorithm enhances the accuracy and effectiveness of the optimization process, filling a crucial research gap in sustainable building design. Secondly, the study conducts a comparative analysis between the DFFA algorithm and other existing approaches, including EPO, LOA, MVO, and FFA. This analysis demonstrates the superiority of the DFFA algorithm in terms of overall cost and energy efficiency. By highlighting the advantages of the DFFA algorithm over other methods, this study further establishes its novelty and effectiveness in achieving sustainable building design goals.

### 1.4 Questions and hypotheses

To provide a clear research direction and facilitate understanding of the research objectives, we have stated the research questions and hypotheses below.

Questions:

− How can the Developed Optimization Algorithm of Farmland Fertility (DFFA) be effectively applied to minimize energy consumption and construction expenses in the design of sustainable buildings?
− What are the comparative benefits of the DFFA algorithm compared to other approaches (EPO, LOA, MVO, FFA) in terms of reducing energy consumption and optimizing building design costs?
− How does the utilization of the DFFA algorithm contribute to improved natural ventilation and interior lighting in sustainable buildings?
− What is the extent of the cost reduction achieved by implementing the DFFA algorithm compared to the initial design, and how does it impact the overall energy efficiency of buildings?

Hypotheses:

− Increasing the surface area of the glass curtain wall and total window space through the optimization process using the DFFA algorithm will lead to noticeable enhancements in natural ventilation and interior lighting within sustainable buildings.
− Despite similar window opening measurements across different optimization methods, the DFFA algorithm will outperform other analyzed procedures in terms of overall cost reduction and energy efficiency.
− The DFFA algorithm will yield desired results within a reduced count of iterations, thereby substantially cutting down the optimization time in contrast to simulation software like TRNSYS and EnergyPlus.
− The utilization of the DFFA algorithm in sustainable building design will lead to cost savings throughout the lifecycle of the building, including reduced energy consumption, operational expenses, and maintenance costs, resulting in improved economic feasibility and return on investment.

The subsequent sections of this study comprise several sections, including:

Materials and Methods: This subdivision extensively defines the materials, methodologies, and authentication process of the Developed Farmland Fertility Optimization Algorithm (DFFO). It specifically focuses on optimizing building envelope parameters, ensuring reliability through rigorous testing and validation, while outlining the objectives and constraints of the optimization challenge.

DFFO Algorithm in the Designing of the Optimization Process: This section explores the practical application of the DFFO algorithm in designing the optimization process. It explains how the algorithm is integrated into the overall building design workflow to minimize energy demand and construction expenses.

Comparative Evaluation: In this section, a comparative evaluation is provided, analyzing the effectiveness of the DFFO algorithm in contrast to alternative existing approaches. It compares the results obtained through the DFFO algorithm with those achieved using methods such as EPO, LOA, MVO, and FFA.

Conclusions and Future Works: The concluding section summarizes the main discoveries of the research, emphasizing the advantages of the DFFO algorithm in energy conservation and cost optimization in sustainable building design. It also highlights potential directions for future research.

## 2 Materials and Methods

In the present study, we employ a Developed Farmland Fertility Algorithm to address the optimization problem concerning the envelope structure of an office building. The following items are considered as the primary decision variables: the number of windows, roof material, glass curtain wall ratio, glass curtain material, window glass material, window length and width, canopy board length and width, and wall material. Through the optimization process, we aim to obtain the optimal values for both the required envelope energy load ($env_{L}$) and the lower envelope energy cost ($env_{C}$). Consequently, the Developed Farmland Fertility Algorithm (DFFA) is regarded as an effective strategy for tackling such problems. In this building envelope optimization scenario, the specified $env_{L}$ is assumed to be acceptable while minimizing $env_{C}$. The architectural facades of the office building are illustrated in Fig. 1.

**Fig. (1):** The architectural facades of the office building.

The variables utilized in this study encompass the type of solar shading panel, the walling material, the ceiling material, the glass curtain wall material, the solar shading panel material, the length of the sunshade board, the window glass material, the quantity of windows, and the dimensions of the window (length and width). Three variants of sunshade boards are considered which are distinguished by their characteristics: $W_{w}$ (window width), $W_{l}$ (window length), and ${Sb}_{l}$ (sunshade board length). The case study locations in this research consist of Guangzhou and Taiyuan in China's Guangdong province.

Equation (1) [21] represents the envelope energy cost ($env_{C}$):

(1) $$env_{C}=A_{wa}\times UC_{wa}+A_{wg}\times UC_{wg}+A_{r}\times UC_{r}+A_{sb}\times UC_{sb}+A_{gc}\times UC_{gc}$$

where $A_{wa}$, $A_{wg}$, $A_{r}$, $A_{sb}$, and $A_{gc}$ represent the respective areas of the wall, window glass, roof, sunshade board, and glass curtain (m^2^). $UC_{wa}$, $UC_{wg}$, $UC_{r}$, $UC_{sb}$, $UC_{gc}$ indicate the unit costs of the wall, window glass, roof, sunshade board, and glass curtain (RMB/m^2^). The mathematical equation of the required envelope energy load ($env_{L}$) is as follows:

(2) $$\begin{array}{c} env_{L}=-20370+0.033\times D_{h}\times C_{hl}+Y_{ihg}\times 2.010+1.079\times \sum_{j=1}^{4}{C_{ing}}_{zj}\times I_{h_{j}}\\ \text{where},Y_{ihg}=Y_{ca}\times 13.5 \end{array}$$

here $D_{h}$ represents the annual degree-hours determined by the monthly mean temperature (kh/y). The thermal transmittance of the building envelope (W/m^2^K) is defined as $C_{hl}$. The yearly internal heat acquisition (Wh/m^2^y) is denoted as $Y_{ihg}$. The coefficient of insolation gain on the z-building envelope orientation is indicated by ${C_{ing}}_{zj}$. The isolation hours (Wh/m^2^y) are represented by I (h_j). The annual cooling air-conditioning hours (h) are specified as $Y_{ca}$, and achieved as below [22]:

(3) $$\begin{array}{c} Y_{ca}=1611+118\times \theta_{i}-3.1\times \theta_{i}^{2}\\ \text{where},\theta_{i}=13.5/C_{hl} \end{array}$$

where $\theta_{i}$ indicates the enhancement in the mean temperature of the room (K) [22]. The following equation defines the thermal transmittance of the building envelope ($C_{hl}$):

(4) $$C_{hl}=(1.011+\;TH_{w}\times A_{wa}+TH_{r}\times A_{r}+TH_{gc}\times A_{gc})/T_{acf}$$

where the wall thermal conductivity, roof thermal conductivity, and glass curtain thermal conductivity (W/m^2^ K) are represented by $TH_{w}$, $TH_{r}$, and $TH_{gc}$ respectively [23]. $T_{acf}$ relates to the overall air-conditioned floor spaces in the building's periphery regions spaces in the building's periphery zones (13139.52 (m^2^)). The window's sunshade coefficient ($W_{sc}$) is defined as below [24]:

(5) $$W_{sc}=f\left({Dr}_{s},T_{sb},O\right)$$

where ${Dr}_{s}$ indicates the depth rate of the sunshade (%), $T_{sb}$ determines the kind of sunshade board, O indicates the orientation. The north orientation (N), south orientation (S), east orientation (E), and west orientation (W) are denoted by orientations I, II, III, and IV, respectively. The mathematical equation of the insolation coefficient gain on the z-building envelope orientation (${C_{ing}}_{zj}$) as follows:

(6) $${C_{ing}}_{zj}=\left(W_{sc}\times \eta \times A_{wg}+0.035\times TH_{w}\times A_{wa}+0.035\times TH_{gc}\times A_{gc}+0.035\times TH_{r}\times A_{r}\right)/T_{acf}$$

where the wall thermal conductivity, roof thermal conductivity, and glass curtain thermal conductivity (W/m^2^ K) are represented by $TH_{w}$, $TH_{r}$, and $TH_{gc}$ respectively. $T_{acf}$ relates to the overall air-conditioned floor spaces in the building's periphery regions spaces in the building's periphery zones. The window's sunshade coefficient is defined by $W_{sc}$. The depth rate of the sunshade is obtained as below:

(7) $${Dr}_{s}=\left\{ \begin{array}{c} \frac{Sb_{l}}{W_{w}}+\frac{Sb_{l}}{W_{l}}\;\left(G:T\;1\right)\\ \frac{Sb_{l}}{W_{w}}\;\left(H:T\;2\right)\\ \frac{Sb_{l}}{W_{l}}\;\left(V:T\;3\right) \end{array}\right.$$

where the width of the window (m) is described by $W_{w}$, the length of the sunshade board (m) is specified by $Sb_{l}$, the length of the window (m) is denoted by $W_{l}$. The letters V, H, and G are used to express vertical, horizontal, and grid sunshade boards [19].

The details of the simulation process are given below:

The information utilized in the simulation for the optimization of building envelopes would have been procured from diverse origins. These sources encompass architectural drawings, blueprints, and CAD models, which are employed to collect building specifications, such as dimensions, floor plans, and design intricacies. The material properties of various building components, such as wall materials, window glass, roof materials, sunshade boards, and glass curtains, have been sourced from technical specifications and building material databases. Climate data, which encompasses temperature variations, solar radiation levels, and insolation hours, holds paramount significance in the evaluation of the energy efficiency of the building envelope. The information presented in this investigation has been procured from diverse sources, including meteorological databases, weather stations, and climate models. Energy simulation software (Energy Plus) has been employed to assess the parameters of energy load. The aforementioned data would provide significant insights into the current energy consumption patterns, thereby facilitating the refinement of more accurate modeling methodologies. The data about costs, which is essential for the computation of envelope energy expenses, have been obtained from databases containing building costs, and prevailing market rates. The examination would encompass the unit prices associated with wall materials, window glass, roof materials, sunshade boards, and glass curtains.

The employment of the Developed Farmland Fertility Algorithm (DFFA) has been employed to effectively address the optimization challenge of the building envelope. Here's an overview of how DFFA applies:

The initialization phase involves the definition of the optimization challenge, which includes specifying the fitness function (${env}_{L}$ and ${env}_{C}$) and decision variables (such as the number of windows, roof material, and glass curtain wall ratio). The variables would have been assigned initial values or ranges. The process of population initialization involves the creation of a population consisting of candidate solutions that represent various configurations of the building envelope. The fitness evaluation process involved assessing each candidate solution within the population according to the fitness function. The calculation ${env}_{L}$ and ${env}_{C}$ would have been performed by utilizing the above equations and the decision variable values corresponding to each solution. The fittest solutions from the population would have been selected based on their fitness values. A new population is generated through the variation operators, which will be fully explained in the subsequent sections. The fitness assessment is performed, and less fit individuals are replaced with the most fit individuals to update the population. Finally, the optimization process concludes when the termination criterion is met. In the following section, the optimization algorithm is described in full and in detail.

### 2.1 Developed farmland fertility optimization algorithm

*The motivation of the algorithm;* Soil is an essential substance on which the life of many organisms on the planet depends. Different combinations of materials such as silica, sand, fertilizer, and clay form different soils that can be suitable or not for the fertility of agricultural land [25]. Fertile soil consists of suitable compounds and suitable animal dung, in other words, plants can provide nutrients for their growth from it [26]. Hence, farmers do various tests through trial and error to get the right combination of soil. In 2018, Shayanfar et al. [27] employed the stated concept of obtaining the optimal mixture of dirt and introduced a novel meta-heuristic algorithm. The offered technique for solving the optimization challenge in this research is named the FFO (Farmland Fertility Optimization), which is described in the next sections.

*Initialization;* First, the initial population of the algorithm consists of the numeral of sections (s) and possible solutions for them (n) in the agricultural land and is gained as below:

(8) N=s×n

Where, s∈[1,N], which is regarded through trials and errors equal to 2 in this study, and n defines an integer amount.

The decision variables in the algorithm are designed based on the following formula and within a specific range.

(9) $$Z_{ij}={\underline{Z}}_{j}+\left({\bar{Z}}_{j}-{\underline{Z}}_{j}\right)\times \Delta$$

Where, ${\bar{Z}}_{j}$ and ${\underline{Z}}_{j}$, denote in turn the bottom and the upper limits of the $j^{th}$ decision variables and Δ describes a value in the interval 0 and 1 at random.

The parts of agricultural land in this study include the global memory part and three local memory parts (A, B, and C), which are presented in the figure below (Fig. 2). The lowest soil quality is related to section A.

**Fig. 2:** The sectors of the agricultural land.

*Analysis of the soil quality;* Based on the computation of the amount of the objective function about decision parameters, the modality of dirt is acquired as below [28]:

(10) $$Q_{q}=Z\left(aj\right),a=n^{*}\left(q-1\right):n\times s\;q=\left[1,\ldots ,k\right],j=1,2,3,4\;\text{.}$$

The mean amount quality of the parts is obtained from the equation below:

(11) $$Fit_{Q_{q}}=mean\left(all\;fit\left(z_{ji}\right)\;in\;Q_{q}\right)\;i=\left[1,2,\ldots ,n\right]$$

*Renovating the memory;* The renewing approach of the memories of local and global has been implemented at this stage. The saving of the agricultures finest solutions is performed in the memory of local and the saving of the solutions amongst them is done in the global memory. The subsequent equations are stated as the numeral of the finest local and global memories

(12) $$K_{local}=round\;\left(t\times n\right)$$

(13) $$K_{Global}=round\;\left(t\times N\right)$$

Where, t defines a constant in the interval [0.1,1], and $K_{Global}$ and $K_{local}$ describe in turn, the numeral of saved solutions in the global and local memory.

*Variety of quality of soil for any part;* The determination of the quality section is done in this stage and then kept in the memory of local. Likewise, the finest candidate is preserved in memory of the global. To modify the worst-instance outcomes, they have been corrected by merging with the finest-instance candidates. Consequently, the renewed candidates are gained as follows:

(14) $$Z_{new}=h\times \left(Z_{ij}-Z_{MGlobal}\right)+Z_{ij}$$

Where $Z_{MGlobal}$ defines a value in the global solutions at random, and $Z_{ij}$ denotes the worst instance of what is utilized for renewing, and h determines a numeral as follows:

(15) $$h=\gamma \times r_{1}$$

Where γ denotes a value in the interval [0,1] which is a constant, and $r_{1}$ defines a value in the interval [-1,1] at random.

Consequently, the novel renewed parts are attained as follows:

(16) $$Z_{new}=h\times \left(Z_{ij}-Z_{MGlobal}\right)+Z_{ij}$$

(17) $$h=\varepsilon \times r_{2}$$

Where ε denotes a value in the interval [0,1] which is a constant, and $r_{2}$ defines a value in the interval [0,1] at random.

*The compound of the soil;* By obtaining local optimal solutions, ($L_{best}$), agriculturalists search for the best soil compound to determine the global optimal solution. The finest global solution for use in agricultural land to improve soil quality is obtained. The next equation can model this:

(18) $$H=\left\{ \begin{array}{c} Z_{new}=Z_{ij}+f\times \left(Z_{ij}-G_{best}\left(b\right)\right),C>rand\\ Z_{new}=Z_{ij}+r_{3}\times \left(Z_{ij}-L_{best}\left(b\right)\right),o.w. \end{array}\right.$$

Where, the finest global solutions and local solution are represented by $G_{best}\left(b\right)$ and $L_{best}\left(b\right)$, C is in the interval [0,1], $r_{3}$ is an amount between [0,1] at random, the fertility variable of farmland at the beginning is indicated by f and reduces with the iteration approach as follows [29]:

(19) $$\omega =f\times R_{v},{0<R}_{v}<1$$

*Terminal circumstances;* The feasible solutions that are available in the search space are computed in this step. The algorithm ends when the termination criteria are obtained, otherwise, it continues until the finest solution is achieved.

### 2.2 Developed Algorithm of Farmland Fertility Optimization

The important issues raised in the application of the farmland fertility optimization algorithm are its low accuracy and premature convergence in solving several particular issues. In this regard, two novel amendments have been considered in the proposed algorithm. The initial one is executed utilizing the OBL (opposition-based learning) procedure [30]. According to the OBL technique, any probable solution with a particular location likewise has a contrary location [31]. To enhance the exploration sufficiency in the meta-heuristic algorithm, this point of view can be employed. Considering that according to the OBL technique, every solution expresses two locations, the finest location is chosen as the original location of the solution. By supposing $Z_{j}$ as a solution in the interval $Z_{j}\in \left[{\underline{Z}}_{j},{\bar{Z}}_{j}\right]$ and its opposite value ${\tilde{Z}}_{ij}$, the equation is simulated as below [32]:

(20) $${\tilde{Z}}_{ij}={\underline{Z}}_{ij}+{\bar{Z}}_{ij}-Z_{ij}$$

where, $Z_{ij},{\tilde{Z}}_{ij}\in R^{i}$.

In this step, the finest candidate in the interval [$Z_{ij},{\tilde{Z}}_{ij}$] is chosen and saved as a solution and the rest candidates are left out. That means in problems of minimization, if $f\left(Z_{ij}\right)>f\left({\tilde{Z}}_{ij}\right)$, ${\tilde{Z}}_{ij}$ is saved and $Z_{ij}$ is left out and inversely. In the present study, the OBL technique has been deliberated on 30 % of the major primary individuals. The subsequent technique is to employ the map of sinusoidal chaos. Minor changes can also affect chaos theory because it regards very sensitive dynamic systems. Improving the distribution of points in the search space by using this technique is because of the formation of several points with a simpler and higher distribution. Hence, the convergence pace of the algorithm adjusts. The model of the chaos theory is stated in the following equation:

(21) $$Z_{i+1}^{j}=f\left(Z_{i}^{j}\right),j=1,2\text{,}\ldots ,l$$

Where l defines the map dimension, $f\left(Z_{i}^{j}\right)$ indicates the generating function of the chaotic model. The basic parameters in this study are stated below based on the sinusoidal chaos map [33]:

(22) $$\begin{array}{c} {\alpha_{i+1}=\alpha_{i}\times p}_{i}^{2}\;\sin\left(\pi p_{i}\right)\\ {\beta_{i+1}=\beta_{i}\times p}_{i}^{2}\;\sin\;\left(\pi p_{i}\right)\\ p_{0}\in \left[0,1\right],\alpha_{1},\beta_{1}\in \left[0,1\right] \end{array}$$

Below is how to set the parameters for the proposed algorithm in a summary and general way.

Initialization (Equation (8)): The parameter denoting the quantity of sections within the agricultural land is represented by the variable s. Conversely, the variable n is utilized to signify the amount of potential solutions for each section. The parameter space for variable s and subsequently determine an optimal value through a process of iterative experimentation are established.

Decision Variables (Equation (9)): The parameters ${\bar{Z}}_{j}$ and ${\underline{Z}}_{j}$ provide the highest and bottom limitations of the $j^{th}$ decision variable, respectively. The random adjustment made within the boundaries is determined by the amount Δ in the range [0,1]. The parameters are determined by considering the specific range and characteristics of the choice factors.

Renovating the Memory (Equations (12), (13))): The constant parameter t, which lies within the range of 0.1–1, governs the proportion of saved solutions in both the global and local memory. The parameter is adjusted to achieve a compromise between the preservation of varied solutions and the prevention of premature convergence.

Variety of Quality of Soil for Any Part (Equations (14), (15), (16), (17)): The parameters h and ε are determined by the constants γ and $r_{1}$, and γ and $r_{2}$, respectively. These constants exert a notable influence on the extent of adjustment applied to the most severe cases during the memory renovation process, thereby affecting the equilibrium between exploration and exploitation within the algorithm.

Compound of the Soil (Equation (18)): The calculation of the optimal global solution for enhancing soil quality is influenced by the parameters C, f, and $r_{3}$. The term C is used to denote the optimal global solution, while the variable f symbolizes the fertility of farmland. Additionally, the variable $r_{3}$ is a value that is created randomly that falls within the range of 0–1. The composition of the soil is determined by these criteria, as indicated by the ideal solutions obtained.

Terminal Circumstances: The execution of the algorithm is finished by achieving the desired level of solution quality.

The sensitivity of these parameters to the functioning of the algorithm can vary. Diverse values assigned to these parameters might result in varying rates of convergence, a trade-off between exploitation and exploration, and the overall quality of the ultimate solutions. The careful selection and fine-tuning of parameters is of utmost importance to attain optimal performance, considering the unique peculiarities of the optimization problem being addressed.

### 2.3 Authentication of the DFFO algorithm

To authenticate the proposed algorithm, ten benchmark tests are used [34]. The considered test functions include ten different types of functions. Utilizing these functions, the offered developed farmland fertility algorithms capability for utilization can be assessed The name of the functions, mathematical representation, and limitation on search sphare are detailed in Table 1.

**Table 1:** Specification of test functions.

Equation	Function	Range
$F_{1}=\sum_{i=1}^{n}x_{i}^{2}$	Sphere	−100< × <100
$F_{2}=\sum_{i=1}^{n}\left|x_{i}\right|+\prod_{i=1}^{n}\left|x_{i}\right|$	Schwefel 2.22	−10< × <10
$F_{3}=\sum_{i=1}^{n}{\left(\sum_{j=1}^{i}x_{j}\right)}^{2}$	Schwefel 1.2	−100< × <100
$F_{4}=\left\lfloor \left|x_{i}\right|,1\leq i\leq n\right\rfloor$	Schwefel 2.21	[-100,100]
$F_{5}=\sum_{i=1}^{n-1}\left|{\left(x_{i}-1\right)}^{2}+100{\left(x_{i+1}-x_{i}^{2}\right)}^{2}\right|$	Rosenbrock	[-30,30]
$F_{6}=-20\times \exp$$\exp\left(-0.2\times \sqrt{\sum_{i=1}^{n}x_{i}^{2}}\right)-$exp$\exp\left(\left(\frac{1}{n}\right)\times \sqrt{\sum_{i=1}^{n}coscos\;\left(2\pi x_{i}\right)}\right)+20+e$	Ackley	[-32,32]
$F_{7}=\frac{1}{4000}\sum_{i=1}^{n}x_{i}^{2}-\prod_{i=1}^{n}\cos\cos\left(\frac{x_{i}}{\sqrt{i}}\right)$	Griewank	[-600,600]
$F_{8}=\sum_{i=1}^{n}\left|x_{i}\;\sin\sin\left(x_{i}\right)+\frac{x_{i}}{10}\right|$	Alphine 1	[-10,10]
$F_{9}=\prod_{i=1}^{n}\left|\sin\sin\left(x_{i}\right)\sqrt{x_{i}}\right|$	Alphine 2	[-10,10]
$F_{10}=\sum_{i=1}^{n}{\left(x_{i}-1\right)}^{2}+\sum_{i=1}^{n}x_{i}x_{i-1}$	Trid	[-100,100]

EPO (Emperor penguin optimizer) [35], LOA (Lion optimization algorithm) [36], MVO (Multi-verse optimize) [37], and the original Farmland Fertility algorithm (FFA) [27] are analyzed by the mentioned function. The parameter adjustments for the algorithms are represented in Table 2.

**Table 2:** Details of the algorithms used.

MVO [37]	$WEP_{\min}$	0.2
	$WEP_{\max}$	1
	Coefficient(P)	6
EPO [35]	$\vec{A}$	0.5
	Temperature value ($T^{\prime }$)	100
	M	2
	f	2.6
	S	1
	l	1.7
LOA [36]	prides quantity	6
	Proportion of nomadic lions	0.2
	Roaming Proportion	0.5
	Mutation possibility	0.1
	Sex level	0.9
	Chance of pairing	0.3
	Ratio of immigrate	0.6

According to the random value of the initial population, optimization processes cannot often create a globally ideal outcome. Nevertheless, they compute a solution that is approximate to an excellent one rapidly. Consequently, 45 modeling of any function are execute.

SD and AVG values are computed. SD indicates the normal deviation, helps in evaluating the deviation in the findings and AVG indicates the average outcomes for the 45 simulations. According to that the goal of resolving these operations is to minimize the function, lesser mean amounts are preferred. Moreover, variation in any instance should be minimized to the greatest extent feasible. Each of the 45 assessments undergoes a grand total of 200 iterations. The STD and average that were achieved for test functions are detailed in Table 3.

**Table 3:** Outcomes of the developed farmland fertility optimization algorithm compared to other existing algorithms.

Benchmark		DFFA	FFA	MVO	EPO	LOA
F1	AVG	0	3.51	5.43	7.26	4.22
	SD	0	2.94	4.18	6.24	2.45
F2	AVG	3.19	6.73	5.43	5.41	5.82
	SD	2.24	5.62	7.39	5.39	4.31
F3	AVG	0	6.5e-11	5.6e-9	6.22e-10	4.93e-9
	SD	0	0.02	4.9e-7	7.51e-5	6.86e-4
F4	AVG	0	0	7.2e-8	9.32e-7	7.69e-8
	SD	0.01	0.07	5.76e-8	7.43e-8	6.88e-9
F5	AVG	0	4.91	5.73	7.36	4.26
	SD	0	5.16	6.93	7.64	7.71
F6	AVG	0.06	6.25	8.46	9.48	6.94
	SD	0	4.12	4.64	4.84	4.37
F7	AVG	0	6.23	6.73	7.94	9.56
	SD	0.74	2.66	3.78	4.22	3.19
F8	AVG	0.01	0.08	1.61	2.92	2.98
	SD	0.07	1.22	2.65	4.74	5.42
F9	AVG	0	0	1.75	4.86	4.25
	SD	0	0	4.73	8.56	6.21
F10	AVG	0	0.46	4.94	7.66	4.54
	SD	0	0.84	1.08	2.67	2.47

As shown in Table 3, the developed farmland fertility optimization algorithm generates the finest outcomes. Likewise, the deviation in the outcome is minimal when analyzed against the dissimilar procedure utilized for the comparison of function. This represents the modified exploitation and exploration abilities of the offered algorithm.

### 2.4 Definition of the optimization problem

The optimization of the walls in all directions is implemented in this part and the walls in the north, south, east, and west directions are not optimized separately. Primary decision variables and principle data of building are presented in the following table (Table 4):

**Table 4:** The major data of building and primary decision variables.

Orientation (z)	${C_{ing}}_{zj}\times I_{h_{j}}$
Building envelope space (m^2^)	20121.13
All space of floor (m^2^)	66241.22
S	13283.66
N	8548.31
W	7884.82
E	9858.86
$Y_{ca}$ (h)	19887.85
Roof	15137.61
$C_{hl}$ (W/ $m^{2}$ K)	7.76
$D_{h}$ (kh/y)	17,189
$Y_{ihg}$ (Wh/ $m^{2}$ y)	26565.14
$T_{acf}$ ($m^{2}$)	14251.19
$\theta_{i}$ (K)	1.98
$env_{L}$ (kWh/ $m^{2}$ y)	49.86
$env_{C}$ (RMB)	15,328,488

The bounds of width and length considered for the window and the bounds of assumed length for the sunshade board are 1–4 m and 1–3 m respectively. The stuff of the wall, glass curtain, window glass, and roof range from 1 to 22, 1 to 4, 1 to 56, and 1 to 18 respectively. The reference number of the stuff is defined by the noted numbers. To provide a comprehensive description of the method used, Fig. 3 is represented as a complete flowchart for the entire study. This flowchart visually represents the steps and organization of the methodology, allowing for a clearer understanding of the process.

**Fig. 3:** The flowchart for the whole study.

## 3 DFFO algorithm in the designing of the optimization process

The process of optimization design includes the process of trial and error, which is displayed in Fig (4) and is also described in the following basic steps: a) Initialization of the algorithm variables is carried out. In the first phase, the fitness function is defined as the $env_{C}$ function which corresponds to the required value of the function of $env_{L}$. b) Adjust iteration equal to 1. c) The Pop (population) computation is performed one time. The matrix of probability amplitude is altered to the matrix in which all the elements are either 0 or 1, for the pop-assessing nature. d) The measurement of the fitness function $env_{C}$ is done at the required value of en, then the finest candidate is obtained in the existing individuals. e) The finest solution (FS) is compared with the finest solutions of every previous individual. When FS is more acceptable than the usual optimum solution (OS), FS and its matching candidate ${\text{FS}}_{i}$ replace the OS, and its matching candidate ${\text{OS}}_{i}$ as the renewed OS and ${\text{OS}}_{i}$. Otherwise, the OS and ${\text{OS}}_{i}$ remain as they are. f) Iteration = iteration+1, the iteration of steps a to f repeats until the termination criterion is satisfied and the iteration is greater than the maximum iteration. g) The OS and ${OS}_{i}$ are achieved.

**Fig. 4:** The flowchart of optimization approach.

### 3.1 Outcomes of DFFO algorithm

The architecture map shown in Fig. (1) is subjected to an optimization test. The comparison between the DFFO algorithm method and the EPO, LOA. MVO and FFA methods through their respective curves are shown in the figure below (Fig. 5).

**Fig. 5:** The DFFA optimization process curve compared with EPO, LOA, MVO, and FFA.

The outcomes achieved at the 200th iteration of the optimization procedure signify the completion of the algorithm's endeavors in seeking the most optimal solution for the architecture of the structure's outer shell. At this point, the algorithm has iteratively refined and adjusted the variables involved in the optimization, aiming to minimize the envelope energy cost ($env_{C}$) while satisfying the desired envelope energy load ($env_{L}$). The $env_{C}$ value of 34, 486, 392.6 RMB represents the minimum cost associated with energy consumption among the various configurations that were assessed. This suggests that the optimized building envelope design successfully produced the most cost-effective solution in terms of energy usage. Through meticulous variable selection and adjustment, including the manipulation of factors such as window quantity, roof material, and glass curtain wall proportion, the algorithm effectively achieved a noteworthy reduction in the energy expenditure entailed in upholding the building's thermal efficiency. Concurrently, the optimized design successfully met the prescribed value for $env_{L}$, which was established as 46.8784 kWh/ $m^{2}$ y. This suggests that the arrangement of the building envelope successfully attained the intended energy load, demonstrating effective energy utilization and decreased energy usage for heating, cooling, and overall thermal efficiency. Table 5 displays the ideal amounts for the variables pertaining to the optimization process, aiming to offer a full overview of the optimized building envelope design. This data presents precise information regarding the selected measurements of the building envelope elements that have contributed to the optimal values of $env_{C}$ and $env_{L}$.

**Table 5:** The finest optimum variables’ values by DFFO.

Variable	Value
$T_{sb}$	2.5
The overall area of the window ($A_{w})$ ($m^{2}$)	448.8
Number of windows ($W_{n}$)	116
The ratio of the glass curtain wall ($R_{gcw}$)	0.42
${UC}_{r}$	5.5
${UC}_{sb}$	3.5
${UC}_{wa}$	3.5
${UC}_{wg}$	1.5
${UC}_{gc}$	3.5
$W_{w}$	2.76
$W_{l}$	1.64
${Sb}_{l}$	1.21
$env_{C}$ (RMB)	11486392.6
$env_{L}$ (kWh/ $m^{2}$ y)	46.8784

## 4 Comparative evaluation

*Comparative outcomes of the DFFO algorithm and several alternative optimization techniques;* In Table 6, the optimization outcomes related to the DFF algorithm method and some other algorithms are presented.

**Table 6:** The optimization outcomes of DFFA and different optimization algorithms.

Variable	EPO	LOA	MVO	FFA	DFFA
$A_{w}$	426.8	386.4	411.8	438.6	438.8
$W_{n}$	132	161	119	121	106
$R_{gcw}$	0.31	0.38	0.39	0.39	0.42
${UC}_{r}$	15	12	13	8	6
${UC}_{sb}$	5	22	16	7	4
${UC}_{wa}$	7	11	14	5	4
${UC}_{wg}$	32	27	18	6	2
${UC}_{gc}$	6	2	5	3	4
$W_{w}$	2.26	1.69	1.92	2.41	2.76
$W_{l}$	1.67	1.69	1.66	1.65	1.64
${Sb}_{l}$	1.31	1.16	1.36	1.26	1.21
$env_{C}$	12684255.2	11988322.5	10822386.7	10,583,946	10286392.6
$T_{sb}$	3	4	4	3	3
Iter*	136	148	85	79	50

(*Iter: iteration number for convergence).

Based on the presented results, it is evident that the lowest value of $env_{C}$ was achieved through the utilization of the developed Farmland Fertility algorithm for solving the optimization problem. Additionally, the use of appropriate materials, such as glass curtain walls, windows, and walls, significantly contributed to optimizing the allocation of the occupied area while still meeting the required environmental performance ($env_{L}$) criteria.

In the presented method, the Developed Farmland Fertility Algorithm (DFFA) demonstrated several advantages. Firstly, it resulted in a larger total window area, indicating a preference for natural ventilation, which can contribute to enhanced indoor air freshness and diminished dependence on mechanical ventilation systems. This aligns with the goal of energy efficiency and sustainable building design. Moreover, the DFFA exhibited a faster convergence rate compared to other methods utilized in similar studies. The downward trend in the number of iterations further supports the higher convergence rate achieved by the proposed algorithm, indicating its efficiency in finding optimal solutions.

Furthermore, by enhancing the $R_{gcw}$ value in the DFFA algorithm, the interior lighting conditions were improved. This suggests that the algorithm successfully considered the balance between energy efficiency and occupant comfort, enhancing the architecture of the structure envelope to maximize natural daylighting while minimizing the need for artificial lighting.

In terms of cost, the presented method demonstrated significant cost savings. The overall price was reduced by 39 % compared to the original design, indicating the economic advantages of the optimized building envelope configuration. By considering factors such as construction materials, window types, and the appropriate utilization of glass curtain walls, the proposed method achieved a more cost-effective design while still meeting the required energy standards.

To reach $env_{C}$ and $env_{L}$ per unit of envelope area, building expense, and energy load were normalized in all expression techniques to make a comparison between them, and the analysis outcomes are presented in Table 7.

**Table 7:** The comparative outcomes of the offered DFFA with alternative approaches.

Variable	EPO	LOA	MVO	FFA	DFFA
$env_{C}$ per unit area	279.65	166.93	228.22	176.386	140.9329
$env_{L}$ per unit area	0.0015	0.0019	0.0016	0.0011	0.0006
The opening rate of the window	–	16.52 %	11.18 %	–	11.22 %

By analyzing the data presented in Tables 7 and it is evident that the suggested method exhibits superior performance than other algorithms in terms of both $env_{L}$ and $env_{C}$ per unit of envelope area. It is important to note that the window opening rate remains approximately the same across all the algorithms, ensuring a fair comparison.

In terms of $env_{L}$, the suggested method demonstrates a lower value in comparison to the other approaches. This indicates that the recommended approach successfully minimizes the environmental impact associated with energy consumption and resource utilization within the building. By optimizing various parameters related to the building envelope, such as insulation materials, window types, and overall design configuration, the suggested method achieves a more sustainable and environmentally friendly outcome.

Furthermore, the suggested method also achieves a lesser value of $env_{C}$ per unit of envelope area. This indicates its superiority with regard to both cost cost-effectiveness and energy management. By employing the Developed Farmland Fertility Algorithm (DFFA), the algorithm used in the suggested method, the building's energy requirements are significantly reduced. This leads to substantial energy savings and improved energy efficiency, ultimately resulting in lower operational costs over the building's lifetime.

Considering the combined effect of the lower $env_{L}$ and $env_{C}$ values achieved by the suggested method, it becomes evident that energy-saving in the building can be better accomplished by utilizing the DFFA algorithm. The algorithm's ability to optimize various aspects of the building envelope design, coupled with its efficient allocation of resources, plays a crucial role in achieving these favorable results.

By obtaining optimal values for both $env_{L}$ and $env_{C}$, the suggested method offers a holistic approach toward sustainable building design. It not only focuses on minimizing environmental impacts but also ensures cost-effective energy consumption. These findings highlight the potential of the DFFA algorithm in supporting energy-efficient and environmentally conscious design decisions within the construction industry.

The existing literature offers a comprehensive examination of the fundamental ideas behind sustainable building design. This study highlights a certain methodology that has the capacity to effectively accomplish objectives related to sustainable building design. The demonstration of the efficiency of the DFFA algorithm serves to showcase the practical applicability of sustainable building design and optimization concepts, thereby making a valuable contribution to the advancement of more efficient and economically viable building designs. In general, both the existing literature and the present study provide support for the objective of sustainable building design and optimization. Collectively, these factors contribute to the continuous endeavor of implementing sustainable building design and optimization strategies that aim to reduce environmental footprints while simultaneously enhancing energy efficiency and cost-efficiency. This study distinguishes itself from existing literature by employing the DFFA algorithm, incorporating empirical evidence from real-world implementation, emphasizing the optimization of building envelope parameters, and making valuable contributions to future research paths. These aforementioned benefits augment the significance of the study and offer significant perspectives that can enlighten and direct actions related to sustainable building design.

## 5 Conclusions and Future Works

The characteristics of a sustainable or green building encompass various aspects such as environmental impact, optimal utilization of resources, and cost reduction throughout the building's life cycle, including design, construction, maintenance operations, reconstruction, and demolition. In the design of green buildings, utilizing building simulation software like TRNSYS and Energy Plus is common practice. However, these software tools require precise input parameters and demand significant time for the simulation process. In this study, the parameters pertaining to the building envelope, such as the number of windows, glass curtain walls, and walls, are optimized to reduce construction expenses. To achieve this, we employed the newly developed Algorithm of Farmland Fertility Optimization (DFFA). Comparative analysis with other approaches such as EPO, LOA, MVO, and FFA demonstrates significant reductions in energy consumption and building design costs achieved by leveraging the proposed algorithm. Furthermore, the DFFA algorithm yields the desired results within fewer iterations. By increasing the surface area of the glass curtain wall and total window space, improvements in natural ventilation and interior lighting are observed. Despite similar window opening measurements across the compared methods, the provided algorithm demonstrated superior performance than others regarding overall cost and energy efficiency. The total cost reduction compared to the initial design amounts to 39 %. Thus, the DFFA algorithm proves to be more effective in conserving energy in buildings compared to other analyzed procedures. In conclusion, this research presents the Developed Optimization Algorithm of Farmland Fertility (DFFA) as a powerful tool for designing sustainable buildings. By optimizing the building envelope parameters, the DFFA algorithm successfully reduces energy consumption and construction costs. The algorithm's efficiency is highlighted by its faster convergence and superior performance compared to other methods such as EPO, LOA, MVO, and FFA. The improvements in natural ventilation and interior lighting achieved through increased glass curtain wall and window space contribute the total energy performance of the structure. This study serves as a valuable case study, demonstrating the applicability of the DFFA algorithm in designing sustainable buildings. Future research in the field of sustainable building design and optimization offers several possibilities for further exploration. One avenue is to integrate additional optimization objectives beyond energy consumption and construction costs. Factors like thermal comfort, quality of indoor air, and environmental impact could be considered to achieve more holistic and comprehensive sustainable building designs. Furthermore, expanding the scope of the study to include different building types and varying climatic conditions would provide a broader understanding of the proposed algorithm's applicability and effectiveness in diverse contexts. This would help establish its generalizability and potential for wider adoption. In terms of methodology, future research could explore the integration of advanced simulation tools and techniques. While this study utilized TRNSYS and Energy Plus, other advanced tools such as advanced energy models, daylighting simulations, or computational fluid dynamics (CFD) analyses could be incorporated to enhance the accuracy and precision related to the procedure of the optimization. To establish the reliability and effectiveness of the Developed Optimization Algorithm of Farmland Fertility (DFFA), further research could undertake extensive validation studies. By comparing the algorithm's predictions with real-world data from existing sustainable buildings, researchers can assess its performance and accuracy in practical applications. Despite the favorable results observed in the optimization of building envelopes, it is crucial to recognize the limitations of the DFFA method in alternative applications. For example, the scalability and complexity of the application may differ when implemented in larger or more involved construction projects, therefore requiring additional research. The algorithm's particular emphasis on optimizing the building envelope necessitates the need for adaptation and exploration to determine its suitability for other facets of building design and optimization, such as HVAC systems or the integration of renewable energy. It is imperative to perform sensitivity analysis to gain an understanding of the algorithm's resilience to various parameter configurations and to assure the production of dependable and consistent outcomes. In addition, it is necessary to conduct further evaluation to ascertain the efficacy of the algorithm in multiple situations, considering variations in climate, building codes, and construction techniques across different geographical regions. The resolution of these constraints via more research and development endeavors will make a significant contribution to the progression of sustainable building design and optimization approaches. This, in turn, will facilitate the implementation of more efficient and economically viable solutions in the forthcoming years.

## CRediT authorship contribution statement

**Chunyuan Yang:** Writing – original draft, Software, Methodology, Conceptualization. **Siyao Yu:** Writing – review & editing, Supervision, Resources, Methodology, Formal analysis, Conceptualization. **Yi Cao:** Writing – original draft, Validation, Software, Resources, Methodology, Formal analysis. **Sama Abdolhosseinzadeh:** Writing – review & editing, Writing – original draft, Validation, Software, Methodology, Data curation.

## Declaration of competing interest

The authors declare that they have no known competing financial interests or personal relationships that could have appeared to influence the work reported in this paper.
